# Effect of Ergonomics-Based Piano Teaching on Teachers' Physical and Mental Health and the Improvement of Sense of Happiness

**DOI:** 10.1155/2022/9174441

**Published:** 2022-03-12

**Authors:** Jian Pi

**Affiliations:** School of Preschool Education of Changsha Normal University, Changsha 410100, China

## Abstract

**Background:**

As a special occupation of human beings, teachers have an important responsibility for society and students. As preachers, all their actions will affect the students. Teachers can be said to be the indicator of students' happy life. According to a survey by educational institutions, more than 90% of teachers believe that work pressure is increasing. 64.2% of teachers have experienced job burnout, and the status quo of teachers' professional well-being is worrying. So we must pay attention to teachers' happiness research. However, based on ergonomics, piano education is a kind of piano education to relieve fatigue and an important way to improve teachers' happiness.

**Objective:**

Using the self-designed questionnaire related to teachers' professional happiness, we investigated piano teachers in universities to understand the status quo of piano teachers' professional happiness, reduce the fatigue of piano teaching, explore the relationship between work fatigue and college piano teachers' professional happiness.

**Methods:**

This study combines qualitative and quantitative survey methods to make a qualitative analysis of the collected literature and survey and, at the same time, to make a quantitative survey of the collected data so as to get more scientific and accurate survey results.

**Results:**

According to the above analysis, this paper puts forward effective suggestions in order to reduce the fatigue of piano teaching and ultimately greatly improve the enthusiasm and efficiency of piano teaching, improve the professional happiness of piano teachers, and promote the effective progress of education.

**Conclusions:**

Through this study, the overall situation of piano teachers' professional happiness in H University is general and the evaluation of piano teachers' professional happiness in H University is mostly at the ordinary level. However, more than half of the teachers do not feel happy and excited at work, and some of them are tired and bored.

## 1. Introduction

Occupation refers to the exertion of individual personality and refers to the realization of human activities in life and sustainable life. The so-called professional happiness means that when human experimenters engage in specific professional activities, they have a sense of psychological satisfaction and joy, which is necessary for life and work. Their psychological activities not only show psychological satisfaction but also reflect their personal ability and give full play to their ability to get a higher sense of experience. At the same time, it is a kind of continuous happy life experience. From the perspective of subjective well-being, individuals are satisfied with the present working life and working state. From the perspective of satisfaction, it is a subjective experience of the working state.

### 1.1. Teachers' Professional Happiness

So far, there is no clear concept of teachers' professional happiness. For teachers, their professional happiness mainly comes from students' evaluation, satisfaction, and achievement in the teaching process, and recognition from colleagues and leaders in the school. Teachers also have their own career plans and goals. If they achieve them, it is also a source of their career happiness [1]. In fact, teachers' career happiness is closely related to students. Teachers, in the process of promoting the development of students, on the one hand, will make their own ability to develop, on the other hand, will also promote the development of students.

So far, there is no clear concept of teachers' professional happiness. For teachers, their professional happiness mainly comes from students' evaluation, satisfaction, and achievement in the process of education, as well as the understanding of school colleagues and leaders [2]. Every teacher has his own career plan and goal. If achieved, it is also a source of professional happiness. In fact, teachers' professional happiness is closely related to students. In the process of promoting the growth of students, on the one hand, teachers improve their ability. On the other hand, they also promote the development of students.

In general, it is a kind of spiritual happiness and satisfaction. It used to be thought that teachers' happiness is teachers' state. In other words, teachers have achieved certain results in life and work, so they often narrow the gap between their goals and understanding. But Durand et al. believe that when he feels happy as a teacher, his contribution is precious [3]. This is a model that benefits both sides. Mastering this sense of happiness is helpful for teachers and students to promote each other. As for the definition of teachers' professional happiness, Appannah and Biggs pointed out that this is their inner satisfaction in their work and life, and they have been realizing their ideals and goals [4], and, in this process, continue to play the greatest enthusiasm, to improve ability, and professional level of themselves [4]. They have been recognized and evaluated by all sides and received more joy and thanks. In this paper, this study adopts the definition of Mr. Wang.

### 1.2. Theoretical Basis of Teachers' Professional Well-Being

Subjective well-being is often defined in the field of western psychology. The focus of this definition is mainly related to the interaction between the internal environment and the external environment. The purpose is to investigate the influence of human personality factors on the social environment and the relationship between subjective well-being and some things in objective reality [5]. How people treat all kinds of personalities, reactions to things, and attitudes in all kinds of environments will affect their subjective well-being. This is the key research content in the field of western psychology. Through the study of subjective well-being, we can know the main source of happiness by studying people's various experiences of happiness. From the existing research results in the field of psychology at home and abroad, many different theories in the field of subjective well-being have been developed [6]. Based on these, many theoretical branches have been expanded. These theories discuss and analyze subjective well-being from different angles and draw some corresponding conclusions. It lays a specific foundation for the subjective well-being theory of University piano teachers, provides a lot of useful theoretical basis and information, and points out the direction for the follow-up research.

#### 1.2.1. The Impact of Career Goals on Well-Being

As we all know, people's subjective well-being is closely related to a variety of people's personality, quality, environment, emotional state, and career goals. Therefore, the supporters of goal theory believe that personal career goals will have a great impact on career happiness, but also related to the personal environment, development direction, future, feelings, and other factors [7]. When each career goal is achieved, these factors are closely related. Then, in order to obtain personal subjective happiness, we must look forward. On the contrary, if an individual fails to achieve his or her goals, it will lead to a more negative emotional experience. Because different goals have different effects, the reasons for subjective well-being vary from person to person.

#### 1.2.2. Theoretical Basis of Pedagogy

Life education theory is a good theoretical method. Its supporters believe that education is to cultivate people who can enjoy happiness, obtain happiness, understand happiness, and inherit happiness. Therefore, for teachers, students usually need to feel the happiness of learning. Happy student learning and happy teacher education are important channels and information sources for teachers to obtain professional happiness [8]. In a sense, teachers' happiness is the premise and foundation. Of course, different teachers have different levels of happiness because of their different morality and wisdom. Therefore, to make every teacher have a professional sense of happiness, we must constantly train and educate teachers to form a good moral character and realize the cultivation of wisdom [9]. Of course, all of these need to constantly pay attention to and improve the happiness level and professional level of teachers so that piano teachers can harvest the happiness of being a teacher.

Life education theory is used to criticize the neglect of life in modern education. Therefore, it is gradually formed and based on this continuous development. The theory of life education pays special attention to respecting life and pursuing life happiness. Life theory has the function of foresight. It may become a procedural theory, guiding teachers and students to pursue happiness has good traction [10]. The goal of this theory is to let teachers and students understand that the pursuit of happiness education is the common ideal and topic of teachers and students. At the same time, it also tells us that the pursuit of happiness, whether teachers or students, is the result of human nature. However, the premise of realizing teachers' professional happiness is the process of life education. Because people's life is the most important, so all this is based on cherishing life and promoting the good growth of personality. Otherwise, it is difficult for teachers and students to get happiness [11]. And it does not make sense. Therefore, for University piano teachers who want to achieve professional happiness, our teachers must adhere to the pursuit of happiness, and the pursuit process is based on the concern for life.

### 1.3. Overview of Ergonomics

Ergonomics includes human physiology, anthropometry, physiological anatomy, biomechanics, medicine, psychology, environmental science, management science, humanities, engineering science, etc., not only in the industrial sector but also in the research of work space, posture, seat, pedal work, operation method, workload, safety, working environment, work schedule, information operator, etc. In addition, it can also provide the design of management mode, the size parameters of “human” in industrial design, the reasonable scientific basis of “object,” and the design guide of “environmental factors” [12]. The main research content can be summarized as the research of humans, including the physiological and psychological characteristics of humans, through the research of humans to solve the relationship between human and machine adaptation problem, to make workers healthy, comfortable, safe, and efficient in operation. Information communication design of the man-machine system, information exchange between man and machine, and reasonable consideration of environment are very important, which is very important in industrial design [13]. Therefore, in the design of the man-machine system, in order to meet the needs of man-machine, the functions of man and machine should be allocated reasonably. Workplace design includes the improvement of the workplace environment and the overall design of the workplace. Appropriate jobs can not only alleviate people's fatigue but also greatly improve work efficiency. In order to ensure the security and reliability of the system, the system security design not only greatly reduces the error rate but also meets the needs of society [14]. The overall efficiency of the system is designed by improving the operation method, optimizing the production or service process, and comprehensively improving the overall efficiency of the man-machine system. The main research methods are observation and investigation (including systematic observation and analysis, investigation, measurement, and recording), experimental method, graphic model method, and simulation method.

### 1.4. Research on Work Fatigue

Work fatigue is a physiological phenomenon that can be recovered through proper rest and adjustment. Due to the work itself, people's sports ability is temporarily reduced. A thorough exercise is a special form of burnout. That is to say, when you are tired, keep exercising until you cannot maintain the normal operation of your body [15]. The causes of work fatigue vary with the degree and place of occurrence. Generally speaking, the symptoms are weakness, hand tremor, waist pain, lower limb pain, yawning, carelessness, loss of memory, lack of thinking agility, etc. Bakker analyzed the executive control ability of piano staff before and after exercise fatigue and compared it with college students who did not receive professional training [16]. The results show that the executive control function of piano instructors and nonprofessional piano education and training students has been improved after work fatigue, and professionals show better executive control function. Yu Shuang's animal experiments show that job burnout may lead to poor learning ability and memory. In order to explore the mechanism of the brain regulating job burnout, Petrou et al. studied the brain function activities of seven healthy male college students before and after a thorough exercise of power bicycle and observed the active exercise in the brain field in the random running stage [17]. Through the use of whole-brain functional magnetic resonance imaging (fMRI) technology, it was found that there was no significant difference in the active parts of the brain before and after work fatigue in the execution stage of random movement, but the number of lines and thalamus in the active nucleus of the brain decreased, and gradually weakened. Tims's research is aimed at 800 m piano teachers [18]. Compared with quiet time, the connections between the primary motor area and cerebellum, somatosensory motor area and cerebellum, hippocampus/parahippocampal gyrus, and cerebellum became weaker after increasing exercise fatigue. At rest, the brain of the subjects formed a stable network system centered on the cerebellum, and the connection function decreased due to burnout and boredom. In short, there are differences in the effects of physical fatigue caused by piano teaching on psychological cognition, which may be related to exercise program, observation place, and detection method.

## 2. Methods

### 2.1. Participants

Based on the principle of research convenience, the piano teachers in H County colleges and universities are selected as the investigation object.

### 2.2. Process

In this study, 190 questionnaires were issued and 190 were recovered by random sampling. The recovery rate is 100%. Among them, 180 effective questionnaires were used, and the effective rate was 94.7%.

### 2.3. Research Design

Master the basic information of teachers such as gender, position, school type, school year, region, and income. There are 10 questions in this questionnaire, and there are several alternative answers after each question. Choose the answer that is consistent with the actual situation and the answer consistent with the situation of yourself. This paper uses the questionnaire of Andrews and wig from foreign countries to measure the overall occupational happiness of teachers [19]. The questionnaire has been evaluated highly internationally, and its reliability and appropriateness reach about 0.7. In this paper, the use of this intuitive graphic option avoids text deviation and improves the accuracy of the survey.

In order to promote the correctness of the investigation, this questionnaire specifically raises 30 specific questions and provides some answers to certain factors so as to better investigate the factors affecting the career happiness of university music teachers [20]. That is, it is divided into complete consistency, more consistent, unclear, no complete consistency, and complete inconsistency. The questioner uses the interview method to ask the teacher's occupational happiness question. In order to supplement the investigation of the influencing factors of the teacher's occupational happiness, let the teacher talk about his own ideas and suggestions so as to obtain a more accurate analysis.

### 2.4. Data Analysis

In this survey, the collected question list will be counted and processed scientifically through Excel and SPSS11.0 and analyzed and discussed by the analysis and processing of the collected data. Finally, based on ergonomics, the paper explores the relationship between alleviating the burnout of piano guidance and the happiness of teachers and makes a deep analysis.

## 3. Results

### 3.1. Analysis of Teachers' Subjective Occupational Happiness

Table 1 shows the statistical results of teachers' subjective occupational well-being towards their current work attitude. On the surface, 4.6% of teachers feel very happy. 34.6% of the teachers were happy, accounting for 39.2% of the total. 13.1% of the teachers were not very happy; 7.3% were unhappy; these two accounted for 20.4% of the total; the remaining 40.4% felt very ordinary.

The image description of teachers' subjective professional well-being survey is shown in Figure 1.

### 3.2. Subjective Factor Analysis

Table 2 shows the statistical results of teachers' response to whether they are satisfied in the workplace. 52.7% of the teachers are dissatisfied and basically dissatisfied in the workplace. In the process of work, 47.3% of teachers are always happy.

As shown in Table 3, the qualifications of music education managers based on ergonomics are not unified. Only three of them are high, and the moderate talents are the main ones, which has a certain impact on the popularization of music culture.

### 3.3. Objective Factor Analysis

In Table 4, “1” refers to teachers under 30 years old, “2” refers to teachers over 45 years old, and “3” refers to teachers over 46 years old. According to the table data, teachers under the age of 30 have the lowest professional well-being, with an average score of 2.286, while teachers over the age of 46 have an average score of 4.571. Second, the occupational well-being of 45-year-old teachers is also very high, with an average of 3.774 years old, but slightly lower than that of teachers over 46 years old.

The image description of the age difference of teachers' professional well-being is shown in Figure 2.

The average score and standard deviation of 180 effective question tables are investigated and analyzed, and a preliminary understanding of the status and characteristics of teachers' working fatigue is obtained. The specific results are shown in Table 5. When answering the questionnaire, use 5 grades of the scoring system. In this system, 1 is absolutely not, 2 is less than once a month, 3 is at least once a month, and 4 is at least once a week at least once a day. From Table 5, we can see that the overall situation of teachers' burnout is more than once a month, which shows that the teachers' burnout is in the middle and high level.

It can be seen from Table 6 that there is an obvious relationship between job burnout, job happiness, and turnover intention. In other words, there is a significant negative relationship between job burnout and job happiness and a significant positive correlation between job burnout and turnover intention. There is a significant negative relationship between job happiness and turnover intention.

Table 6 shows the relationship between job burnout and job happiness. Seven aspects of job happiness (job value, welfare, development prospects, environmental control, self-acceptance, interpersonal relationship, and self-discipline), teachers' scores and the total scores of job happiness and job burnout (physical job burnout, mental job burnout, and emotional job burnout) [21], excluding self-discipline and physical job burnout, teachers' scores and the total scores of job happiness and job burnout (physical, mental, burnout). The relationship between self-discipline and emotional job burnout is not obvious. The rest has a negative correlation, and the correlation coefficient has reached a statistically significant level.

### 3.4. Frequency Table of Ways to Relieve Teachers' Work Fatigue

After classifying the collected questionnaires, the coping methods to reduce work fatigue are summarized and listed in Table 7 according to the frequency.

## 4. Discussion

### 4.1. Job Fatigue Is Related to Teachers' Well-Being and Turnover Intention

Subjective well-being and teachers' turnover intention are the variables of job burnout. Through this study, we can find that the rationality and applicability of the concept of job burnout are influenced by turnover intention. Through the relevant investigation, we found that there is a correlation between teachers' work fatigue and work happiness. Seven aspects (work value, welfare, development prospects, environmental control, self-acceptance, interpersonal relationship, self-discipline) [22] were used to measure job happiness and job burnout (physical burnout, spiritual burnout, emotional burnout). There was no significant relationship between self-discipline and physical burnout except the total scores of self-discipline and emotional burnout. The other factors are negatively correlated with it, and the correlation coefficient is statistically significant.

There is a relationship between teachers' job fatigue and turnover intention. Teachers' turnover intention is related to all aspects of job burnout (physical job burnout, psychological job burnout, emotional job burnout) [23]. The correlation coefficient is statistically significant. There is a negative correlation between teachers' turnover intention and job happiness, between the seven dimensions of job happiness (work value, welfare, development prospects, environmental control, self-acceptance, interpersonal relationship, self-discipline) and teachers' job happiness, and between teachers' turnover intention (physical work fatigue, psychological work fatigue, emotional work fatigue). The correlation coefficient is statistically significant. These results show that job burnout plays an important role in teachers' job happiness and turnover intention [24].

The results show that job burnout has a negative predictive effect on teachers' work, and a positive predictive effect on teachers' turnover intention. Therefore, if enterprises want to improve teachers' job happiness and reduce teachers' turnover intention, they can consider it from the perspective of reducing teachers' job fatigue.

### 4.2. The Professional Well-Being of Piano Teachers Has Significant Differences

The happiness of female teachers is higher than that of male teachers. One of the reasons is that at this stage of society, the demand for men is much higher than that of women. For example, men's wages are higher than women's, and men's working conditions are generally worse than women's. Another reason is the decision and influence of the concept of ancient Chinese traditional culture [25]. In traditional China, it is generally believed that songs are not performed by boys but by girls. Music teachers must also be women. In this way, male teachers are not recognized by society, resulting in their own cognitive bias for their own identity.

Teachers under 30 have the best professional happiness. This is because young music teachers who have just graduated from universities and other roles have become teachers. They have a strong sense of freshness and pride, and they are very enthusiastic. The work of teachers is also very challenging, so it is easy to meet [26].

The higher the level of education, the lower the happiness of teachers. This is because, although the education background of teachers is low, their position is more correct, but they are most concerned about education, and they are also very competent in education business and satisfied with education. Teachers with higher education levels will have more expectations for work, which makes it difficult to get happiness.

Music teachers with the highest professional title have the strongest professional happiness, the second teacher with the lowest professional title, and the teacher with the middle professional title is between the lowest and the highest. For senior teachers, they are conscientious and responsible for their work, have a strong professional ability, have a higher status and understanding in society, and can win the respect and support of students and parents [27]. Wages and welfare are also guaranteed. The most important thing is to treat life, world outlook, and values correctly. That is to say, they have self-knowledge and have higher happiness. Teachers with primary professional titles, who have just taken office, have enthusiasm, are interested in identity changes, have a fresh sense, and their positioning is very correct, so happiness is very high [28]. Instead, if they are intermediate teachers, they have a rich educational experience, but they are older and have a lower sense of professional happiness due to their lazy education. Therefore, schools and governments should create a platform for teachers to improve their education level, constantly strive to inject positive energy into educational activities, and increase opportunities for teachers to continue research and further research.

The smooth development of educational activities is inseparable from teachers, and the educational activities of schools are closely related to teachers. Teachers' high vocational happiness can improve the quality of education to the greatest extent and enable students to grow up comprehensively [29]. In order to reflect the current situation of music teachers' professional happiness in a certain region, this paper will investigate and study the current situation of music teachers' professional happiness in some regions. A survey was conducted in a certain area by questionnaire. It provides the practical foundation for music teachers to obtain professional happiness.

### 4.3. Factors Affecting Teachers' Happiness

From the perspective of the whole social system, it is necessary to improve the economic treatment and social status of teachers. Economic treatment and social status are the important conditions and decisive factors to determine teachers' happiness. In essence, the direct reason for the decline of college music teachers' happiness is the widespread prejudice to overload work and society. Because of the particularity of the professional field, music teachers usually carry out school year music courses separately, and sometimes all music courses in the whole school will be implemented. This will bring great problems and pressure to music teachers in universities.

The current education reform originally put students aside but ignored the cultivation of teachers. The teacher's mood was not carefully considered. Music teacher is an awkward social role among teachers. Although university music teachers are engaged in heavy education and management work, their wages are still low. Needless to say, the benefits of welfare are out of proportion to their work intensity. The material basis determines the superstructure. Similarly, the basic prerequisite for teachers to achieve professional happiness is to have a specific material basis. Therefore, it is very necessary for teachers to create necessary material conditions and corresponding social status. Under the background of the market economy, the economic treatment of teachers must determine their professional happiness. Therefore, the most basic thing to really improve the happiness of teachers is to improve the economic and welfare treatment of teachers.

As a national central government, the education department should increase financial support, and the national government should formulate appropriate measures to ensure teachers' wages and gradually increase teachers' wages and social welfare. We should conscientiously implement the national financial expenditure and narrow the wage gap between teachers in different regions. Government departments continue to guarantee teachers' wages, but local autonomous bodies can also increase financial expenditure in order to increase teachers' wages. A powerful country must strengthen education. In order to strengthen education, it is necessary to increase investment in education. The top priority is to effectively improve teachers' wages and social low level. The state and government should narrow the wage gap of teachers in different regions through policy guarantees, and try their best to narrow the wage and subsidy gap of teachers in county-level cities, big cities, and local areas. To really improve the social status of teachers, so that teachers can feel their own value in the actual educational activities, so as to engage in educational activities at ease.

Society should give music teachers a relaxed environment, more understanding and support, less pressure and reprimand, and a reasonable and fair evaluation. Music teachers are not important to ordinary people. In fact, music teachers in universities are quasi-subject teachers. Music teachers are a troublesome social role among teachers, which generally leads to their low sense of self-existence and professional identity. So what do you say about professional happiness? Society should pay more attention to music teachers, treat their profession fairly, and create a good atmosphere of national trust. Let music teachers find their own professional identity in this atmosphere, urge teachers to regard education as their lifelong career pursuit, and let teachers get countless happiness in this professional education work.

Society needs to set correct and reasonable expectations for teaching staff. Students, families, and society should treat their responsibilities correctly, and teachers should not be excessively held responsible. Because education is not omnipotent, the cultivation of students is formed by the joint action of various facts, not only depending on teachers, but also the society should form the correct direction of teacher evaluation. Therefore, students, parents, schools, and society should have reasonable expectations for teachers, not too harsh. As social media, we cannot exaggerate individual phenomena unilaterally or convey negative energy to society. We must report it actively and objectively. Now some media exaggerate individual teachers' improper behavior to exaggerate the evaluation, which has a very bad impact on the society and even distorts the correct evaluation of teachers. Education reform is vigorously carried out throughout the country. Strengthening publicity, delivering positive energy to society, and forming a correct social atmosphere can gradually change people's wrong ideas.

### 4.4. Suggestions for Relieving Work Fatigue in Piano Teaching

In recent years, enterprises have paid more and more attention to the fatigue of teachers' work, but there is still much room for improvement. Therefore, business operators must take measures to solve these problems, including organizing more outdoor activities, such as going out, dinner, singing, and so on, and establishing effective reward and incentive mechanism. For example, when teachers are praised publicly, part of the bonus is used to comfort them, various bonus systems are set up, and more attention is paid to teachers' life and needs, so that teachers' life trends can be understood in detail. According to the operation of enterprises, within the limited scope of rights, teachers' personal requirements should be properly met, and teachers' interests should be maximized. In the daily work meal, give teachers continuous and reasonable nutrition distribution. Improve the company system, reduce inefficient, repetitive work, and effectively reduce the workload of teachers. The practice of “taking care of teachers” is rooted in the hearts of the people so that teachers can really feel the top-down care and respect, reduce the imbalance of teachers, and improve the happiness of teachers' work. Only when teachers feel the concern and respect of the company, can teachers have the best state in their work and will not bring too much pressure on themselves. This can not only improve teachers' working environment, reduce work fatigue, but also improve enterprise efficiency, increase teachers' sense of happiness, reduce teachers' desire to leave, improve teachers' sense of belonging, improve enterprise culture, and strengthen enterprise unity.

Most of the fatigue of teachers' work is related to their own cognition. Teachers can take various countermeasures to reduce and eliminate the fatigue of work. The general methods used are as follows: a combination of work and rest. Many people believe that when you work, you have to work crazily, and you will indulge in it when you rest and play. In fact, I do not recommend this approach. The best way to live a day is to learn how to combine work and rest. Work should be arranged in a reasonable time and priority, pay attention to rest, not to work in your life to rest. Usually, you can take part in sports activities such as running, swimming, playing ball, walking to ensure the rest time. Whether it is work or play, adults should ensure 7 hours of sleep, preferably not to take up sleep time. The best way to eliminate mental fatigue is to have plenty of sleep. Study work reasonable arrangement. Work and learning are the same, but both need to pay attention to the methods. As long as you have mastered the working methods, you can use less energy to do more, which can improve the efficiency of work and not overwork. Interpersonal communication also needs to be noted that people are social animals, and we can be supported and happy in society. When we have a good interpersonal relationship and work fatigue, chatting with friends and relatives helps to regulate and eliminate mental fatigue. Develop your own interests and hobbies. Whether it is concerned about work or ordinary concern for leisure and entertainment, it needs to be cultivated. It is not possible to be bored with the work of interest. Interest outside of work can also help relieve mental fatigue. When working very tired, you can rest properly, drink water, play games, read books, and distract your attention in order to alleviate the fatigue of work.

## 5. Conclusion

Through investigation and analysis, this study shows that there is no obvious correlation between teachers' professional happiness and their education background, professional title, school type, and educational experience. Teachers' professional happiness is obviously related to gender, age, teaching subjects and grades, school obligations, income, and other factors. In order to change the current situation, there are two main aspects to promote teachers' professional happiness. First, society should make a reasonable and fair evaluation of teachers; schools should take reasonable and objective measures, standardize the system and culture, and use ergonomics to improve teachers' happiness. The other is to improve teachers' own quality and psychological quality and improve their subjective sense of happiness. Although the posture of playing the piano should not be the focus of piano guidance, it is the basis of healthy piano playing. If the piano teachers can guide the learning of piano with the attitude of ergonomics in the basic piano education, reduce the phenomenon of giving up piano due to work fatigue so that more teachers can participate in music practice, improve the quality of music, and then get a sense of happiness. In future research, I will continue to pay attention to the cutting-edge theory of ergonomics and strive to obtain more experimental data to build a framework for the improvement of teachers' well-being.

## Figures and Tables

**Figure 1:** A survey of teachers' subjective professional well-being.

**Figure 2:** Age differences of teachers' professional well-being.

**Table 1:** Questionnaire of teachers' subjective occupational happiness.

Your evaluation of your current job	Frequency	Percentage
Very happy	12	4.60
Relatively happy	90	34.60
General	105	40.40
Less happy	34	13.10
Very unhappy	19	7.30
Total	260	100.00

**Table 2:** Statistics of teachers' subjective feelings about work.

At work, you feel happy	Frequency	Percentage
Totally suitable	11	4.20
More in line with	112	43.10
Doesn't match	106	40.80
Totally inconsistent	31	11.90
Total	260	100.00

**Table 3:** Analysis on the qualification of piano teaching staff from the perspective of ergonomics.

Category	Statistics	Number of people
Age structure	50–59 years old	14
	40–49 years old	7
	30–39 years old	18
	Under 30	15

Title structure	Ortho height	3
	Subtropical high	18
	Lecturer	17
	Teaching assistant	14
	Teaching assistants	3

Academic structure	Postgraduate	23
	Undergraduate	24
	Specialist	9

**Table 4:** Age differences of teachers' professional well-being.

	N	Average	Standard deviation	95% confidence interval of average value		Minimum value	Maximum value
				Lower limit	Upper limit		
1	86	2.286	0.673	2.076	2.495	1.0	3.0
2	108	3.774	0.576	3.615	3.932	3.0	5.0
3	14	4.571	0.534	4.077	5.066	4.0	5.0
Total	208	3.216	1.611	3.017	3.414	1.0	5.0

**Table 5:** Status quo of piano teaching fatigue based on ergonomics.

	Standard deviation (SD)	Average (M)	Number of items (n)	Average score of each question (m)
Physical work fatigue	3.463	20.22	6	3.370
Psychological work fatigue	3.585	19.34	6	3.224
Emotional work fatigue	2.932	18.57	6	3.092
General questionnaire	5.004	58.01	18	3.223

**Table 6:** Analysis of the relationship between piano teaching fatigue and teachers' happiness.

	Physical work fatigue	Psychological work fatigue	Emotional work fatigue	Total score	Turnover intention
Work value	−0.109	−0.213	−0.202	−0.167	−0.297
Welfare	−0.157	−0.243	−0.217	−0.190	−0.352
Prospects	−0.156	−0.17	−0.214	−0.186	−0.217
Environmental control	−0.309	−0.215	−0.296	−0.221	−0.186
Self-acceptance	−0.068	−0.024	−0.232	−0.177	−0.277
Interpersonal relationship	−0.245	−0.212	−0.317	−0.243	−0.408
Autonomy	−0.054	−0.258	−0.061	−0.167	−0.238
Total score for job well-being	−0.321	−0.225	−0.212	−0.245	−0.099
Turnover intention	0.277	0.138	0.355	0.237	

**Table 7:** Frequency of ways to relieve teachers' fatigue.

Solution	Frequency
Do sports	87
Objects (towels, etc.) relieved	35
Drink relief	134
Increase rest time	125
Distract attention from playing games	24
Ease	67
Improve lifestyle (more baths, etc.)	43
School organizes outdoor activities	105
School organization party	98
Schools send out more condolences	76
School lunch increases nutrition	69
Humanization of the school system	129
Others (basking in the sun, etc.)	109

## Data Availability

The datasets used and/or analyzed during the current study are available from the author on reasonable request.
